# GP96 and SMP30 Protein Priming of Dendritic Cell Vaccination Induces a More Potent CTL Response against Hepatoma

**DOI:** 10.1155/2022/2518847

**Published:** 2022-01-07

**Authors:** Rongshi Huang, Jian Pan, Yaoyao Zhang, Qiuhong Qin, Naixia Chao, Tianming Huang, Chengxiao Chen, Feilan Zhao, Guorong Luo

**Affiliations:** ^1^Department of Histology and Embryology, Institute of Preclinical,Guangxi Medical University, Nanning,530021, China; ^2^Department of Histology and Embryology, Institute of Preclinical,Guangxi Traditional Chinese Medical University, Nanning,530001, China

## Abstract

Heat-shock protein (HSP) GP96 is a well-known adjuvant in immunotherapy. It belongs to the HSP90 family. Our previous study demonstrated that DC pulsed with recombinant senescence marker protein 30 (SMP30) could induce cytotoxic T lymphocytes (CTLs) against liver cancer cells in vitro. In this study, SMP30 and GP96 were subcloned into lentiviruses and transfected into DCs from healthy donors. We included six groups: the GP96-SMP30 group, GP96 group, SMP30 group, DC group, empty vector control group, and hepatoma extracted protein group. We used ELISA to detect cytokines and flow cytometry to assess CD80 and CD86 on DCs and the effect of CTLs. Our vector design was considered successful and further studied. In the SMP30 group, DC expresses more CCR7 and CD86 than the control group; in the SMP30+GP96 group, DC express more CCR7, CD86, and CD80 than the control group. Transfected DCs secreted more TNF-*α* and interferon-*β* and induced more CTLs than control DCs. SMP30 + GP96 effectively stimulated the proliferation of T cells compared with control treatment (*P* < 0.01). We detected the cytokines TNF-*α*, TNF-*β*, IL-12, and IFN (*α*, *β*, and *γ*) via ELISA (Figure 5) and verified the killing effect via FCM. Four E : T ratios (0 : 1, 10 : 1, 20 : 1, and 40 : 1) were tested. The higher the ratio was, the better the effects were. We successfully constructed a liver cancer model and tested the CTL effect in each group. The GP96 + SMP30 group showed a better effect than the other groups. GP96 and SMP30 can stimulate DCs together and produce more potent antitumor effects. Our research may provide a new efficient way to improve the therapeutic effect of DC vaccines in liver cancer.

## 1. Introduction

There are limited strategies for the treatment of hepatocellular carcinoma (HCC) [1]. However, DC vaccination is a promising method. As we all know, GP96 is a powerful adjuvant that can stimulate specific immunity. The literature illustrates the important role of GP96 in initiating T-cell immunity [2]. GP96-peptide complexes can be taken up by DCs [3]. Furthermore, DCs express MHC class II molecules and secrete cytokines and chemokines. After maturation, DCs present antigens to T cells and initiate CTL responses [4, 5]. Therefore, based on the adjuvant effects of HSP preparations, vaccination with these preparations has attracted increasing attention in studies of immunotherapy in cancer or infectious diseases. HSP-peptide complexes isolated from intact tumor cells or virus-infected cells or reconstituted by covalent cross-linking or fusion protein strategies are all capable of eliciting potent CTL.

SMP30 was previously shown by our research group to be highly expressed in paracancerous HCC tissues but to be present in low levels in HCC tissues [6]. It is also a potent adjuvant that can induce CTLs against liver cancer cells in vitro.

CTLs respond to antigenic peptides bound to HSPs. Vaccination approaches have even been evaluated in phase III clinical trials for the treatment of human papillomavirus-related carcinoma.

GP96 belongs to the HSP90 family and has been proven to have an efficient stimulatory effect on T cells. We studied SMP30 for a long time and found that it also has the abilities to promote dendritic cell maturation and activation, as described previously by us. Interestingly, GP96 and SMP30 may have potential as novel adjuvants in peptide immunization for the treatment of cancer or infectious diseases. Therefore, we combined these two proteins and determined whether the combination had more potent effects than each protein alone.

## 2. Related Technologies

### 2.1. Cell Lines

HepG2 cell lines, Huh7 cells, and SMMC-7721 cells (Wuhan GeneCreate Biological Engineering Co., Ltd.) were used.

### 2.2. Lentiviral Vectors

A GP96 lentiviral LV5 vector, NM_003299.2., and an SMP30 lentiviral LV8 vector, NM_004683.5 (Shanghai GenePharma Co., Ltd.), were used.

### 2.3. Protein Extraction

HCC tumor tissue was obtained from the Affiliated Cancer Hospital of Guangxi Medical University. Tissues were reviewed and macrodissected by a hepatobiliary pathologist (Prof. Liao). These samples were used as the positive control group.

### 2.4. Immunohistochemistry Assays

We used mouse anti-human HSP90, rabbit anti-human GP96 (Wuhan Boster Biological Technology Ltd.), and mouse anti-human SMP30 (Santa Cruz Biotechnology Inc.) antibodies. Paraffin sections were boiled in 10 mM citrate buffer (pH 6.0) for 20 mins prior to staining (starting dilution: 1 : 50) [7].

### 2.5. Generation of Human Dendritic Cells

Peripheral blood mononuclear cells were isolated from volunteers by Ficoll-Hypaque (Sigma, St. Louis, MO) density gradient centrifugation. Human peripheral blood monocyte-derived dendritic cells were collected, and rhGM-CSF and rhIL-4 were added every two days. The final concentrations were 100 ng/ml and 50 ng/ml, respectively [8, 9]. On day 6, lentiviruses were added for transfection. The experiment included six groups: the DC group (negative control), empty vector group, GP96 + SMP30 group (mixed group), GP96 group, SMP30 group, and extracted protein group (positive control).

### 2.6. Induction of Specific CTLs

T cells were collected by positive selection with CD3^+^ and CD28^+^ beads (Miltenyi Biotec) [10] and then cocultured with the DCs in the above groups in Transwell plates. After 3 days, the CTLs were collected from the bottom wells. T-cell proliferation was compared among the groups. Then, the cells were cocultured with hepatoma cells to verify cytotoxicity.

### 2.7. Western Blot Analysis

The six groups of cells were harvested, and total protein was isolated and quantified. Following sodium dodecyl sulfate-polyacrylamide gel electrophoresis (SDS-PAGE), the proteins were transferred to a PVDF membrane. After saturation, membranes were incubated at room temperature for 2 hours in TBS with 0.1% Tween 20 (TBS-T) containing 5% nonfat dry milk and subsequently incubated with primary antibodies against E6 and E7 (1 : 200 dilution) overnight at 4°C. Peroxidase-conjugated IgG antibodies were used as the secondary antibodies. The protein-antibody complexes were detected using an ECL detection kit following the manufacturer's protocol. *β*-Actin was used as the protein loading control.

### 2.8. Assays for Cytokines

Human dendritic cells were cultured for 6 days and adjusted to 5 × 10^5^ cells/mL in 24-well plates. Then, supernatants from designated wells were harvested after 48 hours for quantification of cytokines, such as interleukin (IL)-12, IL-1, and tumor necrosis factor-*α* (TNF-*α*) or regulated on activation, normal T cell expressed and secreted (RANTES), using ELISA kits (R&D Systems, Minneapolis, MN).

### 2.9. Flow Cytometry Analysis

#### 2.9.1. CTL Effect

Suspensions of effector cells were prepared in fresh culture medium to yield the desired effector : target (E : T) ratios, for example, 40 : 1, 20 : 1, and 10 : 1, when mixed with target cells as described below. Huh7 and SMMC-7721 cells were labeled with a live cell flow cytometry dye (A, green); 1 × 10^6^ cells were treated with 10 *μ*l/ml, washed twice with PBS at 37°C for 20 minutes, and centrifuged to remove excess dye. After coculture for 6 hours, the cancer cells were stained with PI at a concentration of 40 *μ*l/ml and centrifuged at 3000 RPM for 30 minutes, and the supernatant was discarded. The cells were treated at 37°C for 5 hours and detected by flow cytometry.

#### 2.9.2. DC Phenotype

Different groups of cells were collected in 1.5 ml centrifuge tubes and resuspended in different groups of cells after centrifugation with 200 *μ*l PBS. Anti-CCR7, anti-CD86, and anti-CD80 fluorophore-conjugated primary antibodies (1 : 200 dilution of the primary antibody) were added to the corresponding tubes and incubated at 37°C for 1 hour. The tubes were washed again with PBS and resuspended in 200 *µ*l in a dark room.

Then, they were detected by flow cytometry (Beckman CytoFLEX).

### 2.10. Mice Model of Liver Cancer

BALB/c nude mice were housed in the Animal Experiment Center of Guangxi Medical University. The husbandry conditions were an SPF environment with 4–6 mice per cage, and the animals were carefully cleaned and fed. A constant temperature environment (20°C–25°C) with a 12/12-hour light/dark cycle and humidity of 50% ± 5% was maintained. Separate feeding (4 to 6 animals per cage) was performed, and the bedding, cages, drinking water, and food were sterilized and provided according to standard methods. Mice had free access to food and water. All animal breeding was conducted in accordance with the principles and procedures prescribed by the Animal Management and Use Committee of Guangxi Medical University. 30 female BALB/c nude mice which 4-5 weeks old were divided into 6 groups. SMMC-7721 cells (1 × 10^7^ SMMC-7721 cells, 0.1 ml) were injected subcutaneously (s.c.) into the right abdomen of mice. On approximately the ninth day, when the tumor had grown to approximately 100 mm^3^, the modeling was considered successful, and the mice were randomly assigned to the 6 experimental groups: the DC group, empty vector group, GP96 + SMP30 group, GP96 group, SMP30 group, and extracted protein group. Every two days, 0.2 ml bulk T cells were injected into the tumor until the 16th day. Then, the mice were euthanized, and tissue and blood were collected. IL-2 and IFN-*γ* were detected with ELISA and immunohistochemistry assays.

## 3. Results and Analysis

### 3.1. Successful Vector Design

We queried the NCBI website for specific information, and with these details, we designed GP96 and SMP30 lentiviral vectors. The results proved our vector transfection efficiency and stable transfection of the relevant proteins (Figure 1). WB verified that the vectors allowed expression of the GP96 and SMP30 proteins (Figure 2). Therefore, our design was considered successful and further studied.

### 3.2. DC Stimulation Leads to Maturation

Our lentiviral vectors were able to induce the expression of surface markers indicative of DC activation and maturation, such as CD80, CD86, and CCR7 [11]. Research showed that mature IFN-DCs (mIFN-DCs), generated from IFN-DCs primed with an antigen, exhibited elevated expression of CD86 and human leukocyte antigen-DR (minimum criteria for DC vaccine clinical trials) and antigen-presenting abilities comparable to those of mature DCs [12] (Figure 3).

Mature DCs exhibited relatively high IFN-*γ* and IL-1 secretion in the GP96 + SMP30 group (Figure 4).

### 3.3. CTLs Produce a Relatively Potent Effect

SMP30 + GP96 effectively stimulated the proliferation of T cells compared with control treatment (*P* < 0.01). We detected the cytokines TNF-*α*, TNF-*β*, IL-12, and IFN (*α*, *β*, and *γ*) via ELISA (Figure 5) and verified the killing effect via FCM. Four E : T ratios (0 : 1, 10 : 1, 20 : 1, and 40 : 1) were tested. The higher the ratio was, the better the effects were (Figure 6).

By comparing Huh7 and SMMC-7721 cells, we found that SMMC-7721 cells were recognized by these CTLs and showed a more obvious killing effect (Figure 7).

### 3.4. Construction of a Liver Cancer Model and Verification of the CTL Effect

We successfully constructed a liver cancer model and tested the CTL effect in each group. The GP96 + SMP30 group showed a better effect than the other groups (Figure 8).

### 3.5. The In Vivo Killing Mechanism of CTLs

We detected IL-2 and IFN-*γ* after a blood draw and carried out WB and immunohistochemical staining after taking material from mouse tumors. The GP96 + SMP30 group showed a more potent effect on tumors than the other groups (Figures 9–11).

DC vaccination is a good method to treat cancer. However, the effect of DC vaccine in actual treatment is not ideal because the tumor environment suppresses the immune system [13]. Therefore, we need to determine a new strategy. Combining two proteins may be a good method [14]. Studies have indicated that DCs pulsed with recombinant fusion proteins composed of an antigenic fragment and HSP protein can stimulate CTL [15]. The literature also shows that HSP90 can stimulate DCs and induce CTL polarization and activation [16]. A study showed that cross-presenting DCs is highly effective in inducing CTLs capable of eliminating liver cancer [17].

GP96 and SMP30 are both potent adjuvants for DCs and can be used in DC vaccines. However, the combination of these two proteins has not been reported in the literature, and it is unclear whether they are coexpressed in HCC tissue or whether they interact with each other. This study showed that GP96 and SMP30 were coexpressed in hepatocellular carcinoma and might interact with each other and that they act as antigens to stimulate DCs to achieve a better CTL-mediated killing effect. We used lentiviral vectors to transfect DCs. The results showed that this approach was successful. When designing the experiment, we considered that the lentiviral empty vector would also induce CTL to enter the tumor, so we set the empty vector group as one of the negative controls [18].

In cocultures of two kinds of cells, the cells are in direct contact, and cytokines can communicate between the cells to facilitate the next step in separate experiments [19]. Through coculture of DCs and T cells, T cells can be transformed into CTLs. We found different results for each experimental group. Cotransfection of GP96 and SMP30 stimulated CTL proliferation better than other treatments, and flow cytometry demonstrated better cytotoxicity with this combination.

Many preclinical studies indicate that induction of antigen-specific CTLs characterizing viral infections is caused by cross-priming [20]. DC vaccines have been fully explored in vivo and in vitro. CTL response was assessed by IL-2, IFN-*γ*, and expression of CD80 and CD86 [21, 22].

To verify the killing effect, we used different hepatocellular carcinoma cell lines as target cells, such as the HepG2, Huh7, and SMMC-7721 cell lines. We found that experiments with SMMC-7721 cells exhibited a good killing effect, while Huh7 and HepG2 cells showed no effect. We considered this situation to be related to MHC restriction because the SMMC-7721 cell line is derived from Chinese hepatoma cells, the Huh7 cell line is derived from a Japanese patient, and the HepG2 cell line is derived from a Caucasian individual. Both DCs and T cells we collected were derived from Chinese individuals, so the cytotoxic effect of CTLs was dependent on presentation by MHC class I molecules. The results showed that the CTL killing effect increased with increasing doses. The lysate group had the best killing effect (*P* < 0.05) because many antigenic components, including SMP30 and GP96, were included. The GP96 + SMP30 group performed better than the extracted protein group, indicating that GP96 and SMP30 are more suitable as DC vaccines and provide a new strategy.

There are many traditional methods for verifying the killing effect of CTLs, such as Cr51, CCK8, and LDH assay. However, these methods all give false positive or false negative results. According to our flow cytometry analysis, some CTLs were dead, which could easily cause false positive results, so flow cytometry is the best way to analyze the killing effect.

Fluorescence labeling and WB experiments showed that SMP30 and GP96 were successfully cotransfected into DCs, which expressed related proteins. Compared with the vector group and the DC group, each group showed significantly more surface molecule expression on DCs: the mixed group showed promotion of three types (CCR7, CD86, and CD80), the SMP30 group showed promotion of two types (CD86 and CD80), and the lysate group showed promotion of two types (CCR7 and CD80). Among the effects on the molecules, the promotive effect on the expression of CD86 by DCs in the mixed group was significantly stronger than that in the SMP30 group, while that in the SMP30 group was significantly stronger than that in the GP96 group. The expression of CCR7 was highest in the mixed group, reaching 0.38%, which was higher than that in the separate SMP30 group and GP96 group (*P* < 0.05); the expression of CD86 was highest in the SMP30 group and the mixed group, and there was no significant difference between the two. The expression of CD86 in the SMP30 group was higher than that in the GP96 group (*P* < 0.05). CCR7, CD86, and CD80 are markers of DC maturation, indicating that both SMP30 and GP96 induce DC maturation and have a certain synergistic effect. The results showed that cotransfection of DCs with lentiviruses carrying the two protein genes had a stronger sensitizing effect than that of transfection with either lentivirus alone, suggesting that GP96 enhances the presentation of SMP30 and that these two proteins can cooperate within DCs. Heat shock proteins are highly conserved cytoplasmic proteins during biological evolution. Recent studies have found that in addition to being an important molecular chaperone, GP96 can also transfer binding peptides to MHC-I molecules, thereby causing specific CTL responses [23–25]. A study found that compared with the polypeptide alone, HSP protein with mixed peptide and DC incubation produced stronger presentation [26]. In a previous study, we detected that the protein and mRNA levels of HSP90 in liver cancer tissues were higher than those in matched adjacent tissues and normal liver tissues and were related to the clinical pathology of liver cancer [27, 28]. Another preliminary experiment found that GP96 was coexpressed with SMP30 in liver cancer tissues. These results suggest that GP96 in liver cancer patients may improve the ability of DCs to present SMP30. Our experimental results further confirm the above research results.

The day-4 data showed that GP96, SMP30, and the combination of GP96 and SMP30 attacked tumors in the liver cancer model, which had a significant enhancing effect compared with the effect in the control group. The day-12 data showed that SMP30 had a more obvious anticancer effect. The day-14 and day-16 data showed that GP96, SMP30, and GP96 + SMP30 had stronger effects than control treatment and that SMP30 had a stronger effect than the empty vector. These results show that GP96 and SMP30 can be used as liver cancer-specific antigens and have effects in immunotherapy, but currently, they cannot be said to have stronger effects when they are used together to stimulate T cells. It may be that the number of models was not sufficient, and further research is needed. From the ELISA results, GP96, SMP30, and GP96 + SMP30 significantly increased the concentrations of IL-2 and IFN-*γ* in serum in each group, GP96 and SMP30 showed no difference, and GP96 + SMP30 played the strongest role. Therefore, we concluded that GP96 + SMP30-stimulated T cells can have a stronger anticancer effect and that their effect on solid tumors is not the most obvious. It may be that the cytokines in blood cannot fully enter the mass, and further research is needed to determine the mechanism.

We speculate that SMP30 and GP96 work through the JAK-STAT pathway. Since IL-2 signaling can be transduced through 3 different signaling pathways (the JAK-STAT, PI3K/Akt/mTOR, and MAPK/ERK pathways), IL-2 versatility can be achieved [29]. After costimulation with CD28, the optimal activity of IL-2 and these pathways is induced, and IFN-*γ* can also activate multiple signaling pathways, the most common of which is the JAK-STAT pathway [30–32] . The specific pathway or multiple pathways through which C96 is induced by GP96 + SMP30 require further research.

## 4. Conclusions

In summary, this study shows that GP96 and SMP30 are coexpressed in liver cancer and that there may be an interaction between these two proteins. Their combined use as a vaccine to stimulate DCs can achieve improved antitumor effects. This is a new liver cancer immunotherapy strategy.

## Figures and Tables

**Figure 1:** Lentiviral vectors: LV5: GP96 lentiviral vector structure; LV8: SMP30 lentiviral vector structure. (a) GP96-transfected DCs. (b) SMP30-transfected DCs. (a) and (b) show the same location.

**Figure 2:** WB after transfection. (a) Detection of GP96 in 6 groups. (b) Detection of SMP30 in 6 groups. (c) GAPDH as the internal control. The GP96 group expressed more GP96, and the SMP30 group expressed more SMP30, indicating that transfection was successful.

**Figure 3:** Changes in surface markers on DCs. (a) CCR7 expression on the DC surface, ∗ indicates <0.05. (b) CD86, ∗∗ indicates <0.01. (c) CD80.

**Figure 4:** Secretion by transfected DCs. (a) Mature DCs secrete IFN-*γ*. ∗ indicates <0.05 and ∗∗ indicates <0.01. (b) IL-1.

**Figure 5:** Secretion by CTLs. (a) CTL secretion of IFN-*α*, ∗ indicates <0.05. (b) INF-*β*, no significance, suggesting that this cytokine does not have an important role in the CTL effect. (c) INF-*γ*. (d) TNF-*α*. (e) TNF-*β*. (f) IL-12.

**Figure 6:** Detection of CTL killing of SMMC-7721 cells by FCM: each group was tested 3 times. The first quadrant represents the CTL effect. Group 3 was a mixed group, and the data indicated that it had a better CTL response than the single-treatment group (12.07%).

**Figure 7:** Comparison of the CTL killing effect between SMMC-7721 and Huh7 cells. SMMC-7721 cells: the killing effect depended on the dose of CTLs; the more CTLs, the better the effect. Combining two proteins was better than either single protein. Huh7 cells: the killing effect did not depend on the dose of CTLs as the empty vector had a more potent effect.

**Figure 8:** Liver cancer model. (a) The liver cancer model. (b) The GP96 + SMP30 group: tumors had disappeared in some mice on day 4. (c) Tumors harvested from mice. (d) Negative TUNEL staining for apoptosis in the DC group. (e) Positive TUNEL staining for apoptosis in the GP96 + SMP30 group.

**Figure 9:** Tumor growth curve and ELISA results. Curve: the tumor volume in the GP96 + SMP30 group was smaller than that in the protein group on day 4, day 14, and day 16, *P* < 0.05. IL-2: the GP96 + SMP30 group showed secretion of more IL-2 than the other groups, *P* < 0.01. IFN-*γ*: the GP96 + SMP30 group showed secretion of more IFN-*γ* than the other groups, *P* < 0.01.

**Figure 10:** Western blot analysis of tumors. (a) First time. (b) Second time. (c) Third time. (d) Fourth time. 1: protein group, 2: DC group, 3: empty vector group, 4: GP96 group, 5: SMP30 group, and 6: GP96 + SMP30 group.

**Figure 11:** Immunohistochemical staining of tumors. (a) Tumor expressing IL-2 in the GP96 + SMP30 group; the brown cytoplasm indicates positive staining. (b) Tumor expressing IL-2 in the GP96 group; the colorless cytoplasm indicates negative staining. (c) Tumor expressing IFN-*γ* in the GP96 + SMP30 group; the brown cytoplasm indicates positive staining. (d) Tumor expressing IFN-*γ* in the SMP30 group; the colorless cytoplasm indicates negative staining.

## Data Availability

The raw data supporting the conclusions of this article will be made available by the authors, without undue reservation.
